The article "Predicting Parkinson's Disease Progression: Evaluation of Ensemble Methods in Machine Learning" was published in 2022. Journal: J Healthc Eng.

# Predicting Parkinson's Disease Progression: Evaluation of Ensemble Methods in Machine Learning

**DOI:** 10.1155/2022/2793361

**Published:** 2022-02-03

**Authors:** Mehrbakhsh Nilashi, Rabab Ali Abumalloh, Behrouz Minaei-Bidgoli, Sarminah Samad, Muhammed Yousoof Ismail, Ashwaq Alhargan, Waleed Abdu Zogaan

**Affiliations:** ^1^Centre for Global Sustainability Studies (CGSS), Universiti Sains Malaysia, USM, Penang 11800, Malaysia; ^2^School of Computer Engineering, Iran University of Science and Technology, Tehran, Iran; ^3^Computer Department, Applied College, Imam Abdulrahman Bin Faisal University, Dammam 1982, Saudi Arabia; ^4^Department of Business Administration, College of Business and Administration, Princess Nourah bint Abdulrahman University, Riyadh, Saudi Arabia; ^5^Department of MIS, Dhofar University, Salalah, Oman; ^6^Computer Science Department, College of Computing and Informatics, Saudi Electronic University, Riyadh, Saudi Arabia; ^7^Department of Computer Science, Faculty of Computer Science and Information Technology, Jazan University, Jazan 45142, Saudi Arabia

## Abstract

Parkinson's disease (PD) is a complex neurodegenerative disease. Accurate diagnosis of this disease in the early stages is crucial for its initial treatment. This paper aims to present a comparative study on the methods developed by machine learning techniques in PD diagnosis. We rely on clustering and prediction learning approaches to perform the comparative study. Specifically, we use different clustering techniques for PD data clustering and support vector regression ensembles to predict Motor-UPDRS and Total-UPDRS. The results are then compared with the other prediction learning approaches, multiple linear regression, neurofuzzy, and support vector regression techniques. The comparative study is performed on a real-world PD dataset. The prediction results of data analysis on a PD real-world dataset revealed that expectation-maximization with the aid of SVR ensembles can provide better prediction accuracy in relation to decision trees, deep belief network, neurofuzzy, and support vector regression combined with other clustering techniques in the prediction of Motor-UPDRS and Total-UPDRS.

## 1. Introduction

Parkinson's disease (PD) is the second most common and complex neurodegenerative disorder worldwide [1–4]. Both polygenic and environmental factors can cause PD [5]. It is found that, in about 1%–2% of the PD cases (mainly familial), the disease development occurs through a single gene [5]. The main symptoms of PD are bradykinesia (motor features), muscle stiffness, and tremor, along with other symptoms such as sleep disorders (nonmotor features), cardiac arrhythmia, and constipation. Alteration of voice and speech is one of the features of PD. Unified Parkinson's Disease Rating Scale or UPDRS, which shows symptoms' presence and severity, is mainly used in tracking PD symptom progression [6–8]. UPDRS is considered as the well-validated test and the most widely used clinical rating scale for patients with PD [6,9–11]. UPDRS includes 4 sections, in which UPDRS I, UPDRS II, UPDRS III, and UPDRS IV are used to evaluate psychiatric symptoms in PD, activities of daily living, reliable motor symptoms measured in PD recognized by physical exam, and complications of treatment [10]. In many studies, this scale is considered based on Total-UPDRS with the range of 0–176 (176 total disability and 0 representing healthy) and Motor-UPDRS which indicates the UPDRS' motor section with the range of 0–108 (108 indicating severe motor impairment and 0 indicating healthy state) [6].

Machine learning (ML) approaches have demonstrated the capability of handling large volumes of medical datasets and presented perceptive directions [12]. The use of ML-based tools could enhance the safety of individuals [13–15], enhance the quality of medical care [16–18], minimize the costs of medical care [19–21], and support physicians' efforts by manipulating big data of patients' records. ML approaches have been broadly utilized for disorders' classification and prediction [22–30]. Gadekallu et al. [31] investigated the use of machine learning techniques for the prediction of diabetic retinopathy. The authors used the PCA-based Deep Neural Network (DNN) model using the Grey Wolf Optimization (GWO) algorithm for the classification of the extracted features of the diabetic retinopathy dataset. The method was evaluated through the accuracy, recall, sensitivity, and specificity evaluation metrics and compared with the support vector machine (SVM), naïve Bayes classifier, decision tree (DT), and XGBoost. Overall, their method achieved higher accuracy compared with the SVM, DT, and XGBoost techniques. Bhattacharya et al. [32] developed a method for the classification of imbalanced multimodal stroke dataset. The authors implemented the Antlion optimization algorithm on the DNN model to select optimal hyperparameters in minimal time consumption. A positive aspect of their method was that it consumed only 38.13% of the training time on the stroke dataset. An artificial neural network is among the most significant approaches for disease classification and prediction [33–38]. Referring to Berner [39], clinical decision support systems (CDSSs) are special tools that are developed to aid medical specialists in their decision-making, considering particular disorders or diseases. ML approaches can be utilized for designing effective CDSS [36] to aid medical specialists in reaching accurate and timely predictions. CDSSs designed using machine learning approaches have played a significant part in evaluating the existence or the severity of the disease.

In machine learning methods, unsupervised approaches are used to lower the dimensionality of data, which allows the detection of the disease. Besides, these approaches allow manipulating the data, removing the noise from data, calculating the similarity, and segmenting the data [40]. On the other hand, supervised learning approaches are used to enable the final classification, prediction, and diagnosis of the disease [41]. While ML has proven its benefits, the effective deployment of ML needs a great effort from human specialists, considering that no particular approach can present acceptable results in all possible scenarios [12]. Although clinical data are available to researchers to explore, the lack of experience to handle big sources of data might restrict the optimum utilization of these sources. Besides, even though several approaches have been used in disease prediction using various real-world medical datasets, the choice of the deployed approach should consider enhancing the accuracy of the prediction and minimizing the time of computation [42].

The goal of this paper is to present a comparison of machine learning approaches for remote tracking of Parkinson's disease progression. The comparative study is based on clustering and prediction learning approaches. To further improve the accuracy of UPDRS prediction, this study uses ensemble learning in the final stage of the proposed method. Ensemble learning approaches have proven to be effective in prediction tasks [25]. Few studies have incorporated ensemble learning approaches for the development of the diseases diagnosis systems [43], [44]; [45]. Further investigations are needed for the effectiveness of these approaches in UPDRS prediction. Accordingly, we use ensembles of support vector regression and different clustering techniques for PD data clustering. The results are then compared with other prediction learning approaches, deep belief network (DBN), support vector regression, multiple linear regression, and neurofuzzy techniques.

The rest of this paper is organized as follows. We introduce a summary of related works on Parkinson's disease in Section 2. In this section, the results of previous works are discussed. In Section 3, we introduce a new hybrid method for PD diagnosis. In Section 4, we present the method evaluation through a PD dataset. Finally, we present the conclusion and recommendations for future study in Section 5. To simplify, a list of abbreviations we used in this research is presented in Table 1.

## 2. Related Work

Previous literature has presented several approaches that allow PD detection, classification, and severity prediction. In Table 2, we present these studies along with the adopted approaches in each study. In the following, we will introduce a summarization of the up-to-date researches in this field.

Prashanth et al. [68] concentrated on utilizing nonmotor signals in the early diagnosis of PD by deploying NB, SVM, Boosted Trees, and RF. The findings indicated that SVM presented the highest accuracy value of 96.40%. Abiyev and Abizade [69] presented a new methodology for PD diagnosis using FNS and NN. The outcomes of the study presented efficient performance of the FNS compared to other approaches. Singh et al. [70] presented a new approach for PD detection using SVM and presented an overall accuracy of 100%. Çimen and Bolat [60] focused on the vocal signals for PD diagnosis using ANN, MLP, and GRNN. The outcomes indicated that the best performance was achieved using GRNN. Shetty and Rao [71] focused on gait signals in PD diagnosis and other neurological disorders using SVM. The presented approach achieved an accuracy of 83.33%. Nilashi, Ibrahim, and Ahani [61] presented a hybrid methodology by using EM, PCA, ANFIS, and SVR techniques. The findings of the study indicated that the presented methodology can detect the severity of the disease accurately. Ozkan [72] concentrated on vocal indicators by using a hybrid methodology based on PCA with K-NN. The result of the study indicated the robustness of the presented approach with an accuracy of 99.1%. Avci and Dogantekin [62] presented a new methodology for PD detection based on GA, wavelet kernel, and ELM. The findings of the study indicated that the hybrid approach presented better prediction accuracy than other state-of-the-art related approaches.

Three ML methods, namely SVM, NB, and RF, were deployed by Rovini et al. [74] and presented an encouraging outcome with a specificity value of 0.967. The vocal signals of PD were assessed by Pahuja and Nagabhushan [73] by using ANN, K-NN, and SVM. The outcomes of the evaluation indicated that ANN presented the most accurate performance with an overall accuracy of 95.89%. In a study by Nilashi et al. [63], SOM, NIPALS, and ISVR approaches were used in PD prediction and presented a robust performance in forecasting UPDRS while minimizing the time of prediction. Parisi et al. [64] presented a hybrid approach based on SVM (MLP-LSVM). The deployed method presented the highest accuracy in comparison with other techniques for PD diagnosis. Prince and De Vos [65] deployed several approaches for PD diagnosis, focusing on severity detection. The deployed approaches entail LR, RF, DNN, and CNN. Among the used approaches, CNN presented a better prediction accuracy of 62.1%. Another study that concentrated on PD's severity prediction was presented by Zou and Huang [66]. In the deployed method, rTL, LASSO, and ebTL approaches were used, among which ebTL presented the best prediction accuracy.

Grover et al. [67] adopted the DNN for severity prediction among PD patients. The deployed method presented encouraging results with an overall prediction accuracy of 81.66% based on the Motor-UPDRS score. Several supervised approaches were presented by Khoury et al. [59] for PD diagnosis, focusing on gait signals, such as K-NN, NB, SVM, RF, and CART. These approaches were combined with other unsupervised approaches to meet the goal of the study. Among the deployed methods, K-NN, RF, and SVM presented the highest accuracy result. Nilashi et al. [46] presented a new approach based on DL and clustering methods. Particularly, they used DBN and SVR for UPDRS prediction. SOM was used as a clustering method to enhance the prediction accuracy. The method was assessed based on a real-world dataset and the proposed approach of clustering, DBN, and SVR presented predictions' accuracy that outperformed other learning approaches. Ghaderyan and Fathi [47] concentrated on analyzing gait signals for PD detection. The basic method is based on separating various parts of the signal, choosing the most related parts that are utilized to measure interlimb divergence in singular value space. The proposed method presented an average accuracy of 95.59% and 97.22%. Nilashi et al. [75] presented a hybrid approach that utilized the clustering method, SVD, and ANFIS. They indicated that the presented methodology outperformed other state-of-the-art approaches in terms of detection accuracy and minimizing the time of computation.

Ashour, El-Attar, Dey, Abd El-Kader, and Abd El-Naby (2020) utilized the LSTM, focusing on the FOG signals collected from several sensors worn on parts of the body. Besides, SVM and ANN were used in the classification process. Although they achieved an overall accuracy of 83%, one shortcoming related to the size of the data can impact the generalizability of the outcomes. Paragliola and Coronato [48] investigated the performance of hybrid NN, which entails CNN for reducing the dimensionality and LSTM for the diagnosis. The study concentrated on walking patterns by utilizing gait data and presented an accuracy of 95%. Still, the applied methodology focused on binary classification issues, in which the severity of the disease was not explored.

In a study by Mohammed, He, and Lin [53], a CNN model for discriminating PD patients from healthy controls, based on SPECT modalities, was proposed. The model was assessed based on 10-fold cross-validation and presented an accuracy of 99.34%. In a study by Balaji et al. [49], a DL approach based on LSTM was developed for severity classification of the PD and presented encouraging results with an overall accuracy value of 98.6%. De Souza et al. [50] presented a Fuzzy OPF for PD diagnosis. RBM was used to extract the features and outperformed other baseline models. Senturk [51] developed an ML method for PD diagnosis. In this study, SVM was used for the classification task and presented an overall accuracy of 93.84%. De Vos et al. [52] used a novel method to discriminate between PSP and PD by utilizing two approaches of LR and RF. RF presented higher accuracy results compared to LR.

In a study by Goyal et al. [54], a hybrid method for feature extraction that integrates RSSD and T-F algorithms was presented. The deep learning approach, particularly CNN, was utilized in PD diagnosis based on speech impairments. The hybrid method presented accurate outcomes in classifying PD patients (99.37%). Based on handwriting assessment, a study by Xu and Pan [55] adopted an ensemble learning model based on RF in the PD diagnosis. Dimensionality reduction was performed using PCA. The presented approach has an overall accuracy of 89.4%, which outperformed LR and SVM based on the adopted evaluation method. Another study, which concentrated on handwriting indicators, was presented by Ribeiro et al. [56]. The study adopted a PD diagnosis approach based on RNN by utilizing the bag of samplings to measure several compact representations and presented acceptable performance compared to other methods in the literature. Another study that concentrated on handwriting was proposed by Parziale et al. [57] based on CGP. This approach presented an explicit decision measure that was used in the detection of PD. The authors also compared various AI approaches for PD detection and indicated that CGP outperformed these approaches in terms of accuracy. Tsuda et al. [58] adopted an approach based on NNs to distinguish between PD and MSA. The adopted methodology presented an improved recognition of the patterns compared to other approaches.

## 3. Methodology

In the prediction of diseases, ML techniques have proven to be effective [77–79]; [25]; [26]; [61]; [27] [42]. This study uses both unsupervised and supervised learning techniques to diagnose PD through UPDRS prediction. Several approaches that entail clustering, reducing dimensionality, and learning of prediction approaches are used to create the PD diagnoses method.  Figure 1 depicts the proposed method with its main stages. Data preprocessing, dimensionality reduction using PCA, clustering using ensembles of EM, and prediction using ensembles of SVR are all stages of the method that are utilized to predict UPDRS through a set of real-world PD data.

**Step 1 .**

(data preprocessing). As suggested by previous studies, the data is preprocessed [80, 81] to have a more accurate prediction of UPDRS. The goal of data preprocessing in this study is to handle the dataset's null values. In general, we included the preprocessing stage in the proposed method because it is typically completed during the first step of data analysis. The data is then deployed in the data analysis stages, such as clustering and prediction. The datasets are created with null values for method evaluation. Before clustering and classification tasks, these values must be imputed. In this study, SVD is used for missing value prediction.

**Step 2 .**

(data clustering). We use an unsupervised learning technique in this stage for clustering the PD data. The objective of this step was to increase patient record readability through the grouping of patients into different groups. We used ensembles of EM to have a better cluster analysis of the data.

**Step 3 .**

(dimensionality reduction). To remove the noise of data, the PCA method was used in this phase to lower the dimensionality of the data [82]. Multicollinearity has a considerable impact on the accuracy of predictors and is a major issue in the field of disease diagnosis [46]. The accuracy of SVR predictors has been affected by the multicollinearity of the data. We, therefore, use PCA to solve the multicollinearity problem as the most popular technique for noise removal.

**Step 4 .**

(UPDRS prediction). This stage was performed to predict UPDRS according to the input features. In contrast to the previous prediction methods for PD diagnosis, we used ensembles of SVR to perform this task. SVR is trained to build prediction models with training datasets. It is a common practice to seek the advice of several doctors who are experts in the field in various clinical settings. The ultimate decision for a specific therapy is thus normally made through consultation and a combination of opinions of a committee of specialists. Ensemble learning systems serve a similar function in the machine learning context [83]. In general, ensemble learning systems can be utilized effectively in classification and regression problems and provide more reliable predictions than any individual learning model [84]. In fact, several weak hypotheses are combined in ensemble learning systems to form a stronger theory. Note that the success and effectiveness of ensemble learning approaches are heavily dependent on the diversity of the individual predictors that construct the ensemble. The total error can be reduced by combining the output of different prediction models through an algebraic expression (e.g., mean value of the predictions), as the various errors of the prediction models are averaged out.

### 3.1. SVR Ensembles

Cortes and Vapnik [85] developed SVM as a machine learning technique for forecasting problems with the potential to be extensively used as a benchmark. Support vector classification (SVC) and SVR are the two main branches of SVM. SVR performs the prediction of a new sample by training the data with target values. This is done by finding Φ(*x*)  function to map data to a flat space. The SVR can effectively solve complex prediction problems through linear and nonlinear regression. The kernel functions are used to transform the data into a high-dimensional feature space. Radial basis functions (RBF) and polynomial functions are the most widely utilized kernel functions in SVR.

Let us have a training dataset of length  *N*: *T*=(*x*_1_, *y*_1_), (*x*_2_, *y*_2_),…, (*x*_*N*_, *y*_*N*_), where *y* ∈ ℜ and *x*_*k*_ ∈ ℜ^*n*^, *k*=1,2,…, *N*, to model a single output (*y*)   in the original SVR; a linear model formulation is presented as

(1) $$\begin{array}{c} \hat{y}\left(x\right)=\langle w,x\rangle +b, \end{array}$$

where $\hat{y}$ indicates the predicted output, *b* is a bias term, *w* is a weight vector, and 〈., .〉 indicates vector inner product. To solve nonlinear problems, in SVR, it is possible to use nonlinear kernel functions, Φ(*x*), and we have

(2) $$\begin{array}{c} \hat{y}\left(x\right)=\langle w,\Phi \left(x\right)\rangle +b. \end{array}$$

One of the most widely employed nonlinear SVR kernels is radial basis functions. In SVR, to have good generalization performance, weight vector *w* is required to be as flat as possible. Thus, for every data point in the dataset, we need to minimize the norm (.) of *w* as

(3) $$\begin{array}{c} \text{minimize}\frac{1}{2}{\left\|w\right\|}^{2},\\ {\text{subject to y}}_{i}\langle w,\;\Phi \left(x_{i}\right)\rangle -b\leq \varepsilon \langle w,\;\Phi \left(x_{i}\right)\rangle +b-y_{i}\leq \varepsilon . \end{array}$$

To guarantee feasible constraints, slack variables (*ξ*_*i*_,  *ξ*_*i*_^*∗*^) are introduced as well as *ε*-insensitive loss function $L\left(\varepsilon ,y,\hat{y}\right)$. Thus, the following cost function needs to be minimized by estimating the parameters *w* and *b*.

(4) $$\begin{array}{c} \text{minimize}\frac{1}{2}{\left\|w\right\|}^{2}C\sum_{il}^{N}\left(\xi_{i}+\xi_{i}^{*}\right)y_{i}-\langle w,\;\Phi \left(x_{i}\right)\rangle -b\leq \varepsilon +\xi_{i},\\ {\text{subject to y}}_{i}\langle w,\;\Phi \left(x_{i}\right)\rangle -b\leq \varepsilon \leq \varepsilon +\xi \partial_{i}^{*}\xi_{i},\;\xi_{i}^{*}\geq 0, \end{array}$$

where C  is the regularization parameter. The above optimization problem can be solved in its dual through handling the constraints by employing the Lagrange multipliers *η*, *η*^*∗*^,  *β* , and *β*^*∗*^. Thus, Lagrangian (*L*) is presented as

(5) $$\begin{array}{c} L=\frac{1}{2}{\left\|w\right\|}^{2}+C\sum_{i=1}^{N}\left(\xi_{i}+\xi_{i}^{*}\right)-\sum_{i=1}^{N}\beta_{i}\left(\varepsilon +\xi_{i}-y_{i}+\langle w,\;\Phi \left(x_{i}\right)\rangle +b\right)-\sum_{il}^{N}\beta_{i}^{*}\left(\varepsilon +\xi_{i}^{*}+y_{i}-\langle w,\;\Phi \left(x_{i}\right)\rangle -b\right)-\sum_{il}^{N}\eta_{i}\xi_{i}-\eta_{i}^{*}\xi_{i}^{*}. \end{array}$$

In order to find the minimum, the following final problem of quadratic programming results in Karush–Kuhn–Tucker conditions as

(6) $$\begin{array}{c} \text{minimize}\frac{1}{2}\sum_{i-1}^{N}\sum_{i-1}^{N}K_{ij}\left(\beta_{i}-\beta_{i}^{*}\right)\left(\beta_{j}-\beta_{j}^{*}\right)+\varepsilon \sum_{i-1}^{N}\left(\beta_{i}+\beta_{i}^{*}\right)-\sum_{i-1}^{N}y_{i}\left(\beta_{i}+\beta_{i}^{*}\right),\\ \text{subject to}\sum_{i-1}^{N}\left(\beta_{i}+\beta_{i}^{*}\right)=00\leq \beta_{i},\;\beta_{i}^{*}\leq C. \end{array}$$

Here, *K*_*ij*_ indicates the kernel function. Finally, in SVR, the model form in the dual space can be written as

(7) $$\begin{array}{c} \hat{y}\left(x\right)=\sum_{i-1}^{N}\left(\beta_{i}-\beta_{i}^{*}\right)K\left(x,x_{i}\right)+b. \end{array}$$

### 3.2. PCA

Pearson [86] introduced PCA as a statistical technique to simplify the complexity of high-dimensional data. This can be accomplished by the orthogonal projection of the correlated variables into uncorrelated variables. The uncorrelated variables are then known as principal components (PCs).

We tested Pearson Correlation Coefficient (PCC) for the interdependencies in the data. If *y* is the output and *x*_*i*_ is the ith  observation in the dataset, the PCC is defined as

(8) $$\begin{array}{c} R_{\left(i\right)}=\frac{\text{cov}\left(x_{i},y\right)}{\sqrt{\text{var}\left(x_{i}\right)\text{var}}\left(y\right)}\\ =\frac{\sum_{k=1}^{m}\left(x_{k,i}-{\bar{x}}_{i}\right)\left(y_{k}-\bar{y}\right)}{\sqrt{\sum_{k=1}^{m}{\left(x_{k,i}-{\bar{x}}_{i}\right)}^{2}\sum_{k=1}^{m}{\left(y_{k}-\bar{y}\right)}^{2}}}. \end{array}$$

Here, cov  is the covariance and var indicates a variable variance.

### 3.3. EM and SOM Ensembles

#### 3.3.1. EM Clustering

EM is a probabilistic and iterative algorithm that switches between the maximization (*M*) and expectation (*E*) phases in a sequential fashion. In the E-phase, EM calculates the expected value of the likelihood function. In M-phase, however, EM obtains an estimation of the parameters to maximize the likelihood function. The parameters obtained in the M-phase are then used in a subsequent E-phase. This process is repeated until convergence occurs (i.e., it convergences to the final values of the parameters). To perform E-phase for the probabilities calculation of which input in the dataset belongs to which mixture model or cluster, EM performs the following formula:

(9) $$\begin{array}{c} p{\left(m|n\right)}^{t}=\frac{w_{c}^{t}h\left(X_{n},\mu_{m}^{t},\sigma_{m}^{t}\right)}{\sum_{k=1}^{M}w_{k}^{t}h\left(X_{n},\mu_{k}^{t},\sigma_{k}^{t}\right)}, \end{array}$$

where *h* indicates the probability density function of input *X*_*n*_ in the dataset for the cluster *m* with standard deviation (SD) *σ*_*m*_^*t*^ and mean *μ*_*m*_^*t*^ at iteration *t*.

Here, normal univariate, bivariate, or multivariate probability density function may be employed and should be according to the dimensionality of data. In addition, under the constraint ∑_*k*=1_^*M*^*w*_*k*_^*t*^=1,   the allocation of data to mixture models is influenced by a weighting factor *w*^*t*^. Accordingly, performing M-phase, for the maximization of the likelihood to the data, EM needs the following computations for each cluster:

(10) $$\begin{array}{c} \mu_{m}^{t+1}=\frac{\sum_{n=1}^{N}p{\left(m|n\right)}^{t}x_{n}}{\sum_{n=1}^{N}p{\left(m|n\right)}^{t}},\\ \sigma_{m}^{t+1}=\sqrt{\frac{{\sum_{n=1}^{N}p{\left(m|n\right)}^{t}x_{n}-\mu_{m}^{t+1}|}^{2}}{\sum_{n=1}^{N}p{\left(m|n\right)}^{t}}},\\ w_{k}^{t+1}=\frac{\sum_{n=1}^{N}p{\left(m|n\right)}^{t}}{N}. \end{array}$$

The above procedure is repeated by executing *E* and *M* phases until convergence occurs.

#### 3.3.2. SOM Clustering

Kohonen's SOM system is an unsupervised machine learning method. Thus learning method is widely used in the visualization of complex data, image processing, speech recognition, data mining, process control, and diagnostics. Based on the characteristics of features, SOM's algorithm tries to map m-dimensional input vectors *x*_*j*_ to two-dimensional maps. SOM aims to reduce the dimensions of the data, which aids in the understanding of high-dimensional data. SOM by this way can present the data in similar groups. Two layers make up a basic SOM. Input space' nodes are included in the first layer, and the output space' nodes are included in the second layer. SOM's idea is to adjust the nodes to represent the distribution of the data. The nodes represent clusters that reflect the distribution of the data. The SOM algorithm starts by assigning random weights to the variables. SOM algorithm in three main stages is shown in Figure 2.

#### 3.3.3. Cluster Ensembles

A number of various clustering approaches form cluster ensembles to partition the initial dataset and concentrate on the enhancement of the clustering outcomes resulting from a mixture of the results of different clustering. This is performed to overcome the instability of the methods of clustering. The fusion approach begins with the clusters formed during the combination phase and determines the optimal number of clusters in the dataset based on certain predetermined criteria. Next, we describe the cluster ensemble approaches, hypergraph partitioning, and majority voting. They are also called consensus functions.

#### 3.3.4. Hypergraph Partitioning

The cluster label vectors for hypergraph partitioning are transformed into a hypergraph image. In particular, there are vertices and hyperedges in a hypergraph. The clusters are represented in a graph as hyperlinks, whose vertices match the clustered objects. A set of objects that belong to the same group are described on every hyperlink. There are three common functions for transforming the cluster set into the representation of the hypergraph. They are CSPA and HGPA. The CSPA uses a Metis algorithm to induce an association matrix graph and cluster it [25]. A clustering in CSPA refers to a link between objects in the same segment of data and can be employed for measuring the similarity in pairs. Then, the similarity will be deployed to recluster the items in order to generate an integrated clustering. In the HGPA algorithm, the problem of cluster ensembles is viewed as a partitioning issue of a suitably identified hypergraph, which represents the clusters. Minimal cut algorithms are mainly used to control the partition size and to find good hypergraph partitions when they are combined with the proper objective functions.

#### 3.3.5. Majority Voting

In the majority voting mechanism, the cluster that is the one with the most votes is selected. Assume a dataset contains four Parkinson's disease patients (PDP1, PDP2, PDP3, and PDP4), and there are three clustering algorithms (Algorithms 1–3). Assume that Algorithms 1 and 2 have both assigned PDP1 to cluster A, while Algorithm 3 has assigned it to cluster B. Cluster A would then be chosen as the best cluster for PDP1 based on the majority vote.

### 3.4. Imputing Missing Value

In this research, we use SVD for missing values imputation. The procedure for missing value prediction by SVD is provided in Algorithm 2. Five steps are used in the SVD algorithm to predict the missing value in the PD dataset. In the first stage of the algorithm, the data is converted to a dense matrix **B**^*m*,*n*^. In the next stage, we perform a normalization procedure on the **B**^*m*,*n*^. In the third stage of the algorithm, we apply the SVD technique to the matrix produced in the second step. Then, we use matrix *Z* to approximate **Z**_*d*_. In the last step, the missing value is predicted.

## 4. Methods Evaluations and Results

In the first step of our data analysis, EM and SOM algorithms were performed on the PD dataset. We implemented EM and SOM to generate a different number of clusters to have their ensembles for final clustering results. Specifically, we run EM for *k* = 8, 10, 12, and 13 and SOM for different SOM maps, SOM2×3, SOM2×4, SOM3×3, and SOM3×4. The results of EM clustering for 13 (*k* = 13) clusters and SOM clustering for 9 clusters (SOM3×3) are provided in Figure 3. These clusters are then used for ensemble learning to be used in UPDRS prediction by the SVR technique.

SVR was trained through the RBF kernel. The SVR parameters are penalty factor *C* and loss function *ε*, and the parameter for RBF kernel is *γ*. These parameters can have a significant impact on the prediction quality of SVR. The radial basis function is defined as

(11) $$\begin{array}{c} K_{ij}=K\left(x_{i},y_{j}\right)\\ =\text{ exp }\left(-\frac{\left\|x_{i}-y_{j}\right\|{}^{2}}{\gamma^{2}}\right), \end{array}$$

where a single parameter *γ* in (11) indicates the spread of the function.

We used 5-fold cross-validation with a grid search mechanism to select the best parameters of each SVR. In the grid search, *γ* was explored on *γ*∈ [0.01 to 0.1] at an interval of 0.005, loss function *ε* was explored on *ε*∈ [0.0001, 0.002] at an interval of 0.0001, and the penalty factor *C* was explored on C∈ [3, 4.1] at an interval of 0.005. We developed the ensembles on bootstrap samples drawn from the selected data points. The training was repeated 8 times to get 8 SVRs. To measure the performance of the presented methodology, we use several metrics such as adjusted coefficient of determination (*R*^2^), prediction accuracy (PA), Index of Agreement (IA), MAE, and RMSE. Their formulas for *n* observations are shown as follows:

(12) $$\begin{array}{c} RMSE=\sqrt{\frac{\sum_{i=1}^{N}{\left({\text{Predicted}}_{i}-{\text{Observed}}_{i}\right)}^{2}}{n}},\\ MAE=\frac{\sum_{i=1}^{N}{\left|{\text{Predicted}}_{i}-{\text{Observed}}_{i}\right|}^{2}}{n},\\ Index\;of\;Agreement\;\left(IA\right)=1-\left[\frac{\sum_{i=1}^{N}{\left({\text{Predicted}}_{i}-{\text{Observed}}_{i}\right)}^{2}}{\sum_{i=1}^{N}{\left({\text{Predicted}}_{i}-{\bar{\text{Observed}}}_{i}\right|}^{2}\left|+\right|{\left|{\text{Observed}}_{i}-{\bar{\text{Observed}}}_{i}\right)}^{2}}\right]\\ \text{p}rediction\text{ a}ccuracy=\frac{\sum_{i=1}^{N}{\left({\text{Predicted}}_{i}-\bar{{\text{Observed}}_{i}}\right)}^{2}}{\sum_{i=1}^{N}{\left({\text{Observed}}_{i}-\bar{{\text{Observed}}_{i}}\right)}^{2}},\\ R_{adjusted}^{2}=1-\left(1-\frac{\sum_{i=1}^{N}\left({\text{Observed}}_{i}-\bar{\text{Observed}}\right)\left({\text{Predicted}}_{i}-\bar{\text{Predicted}}\right)}{\sqrt{\sum_{i=1}^{N}\left({\text{Observed}}_{i}-\text{Observed}\right)}\times \sqrt{\left({\text{Predicted}}_{i}-\bar{\text{Predicted}}\right)}}\right)\left(\frac{n-1}{n-m-1}\right)\\ =1-\left(1-R^{2}\right)\left(\frac{n-1}{n-m-1}\right), \end{array}$$

where $\bar{\text{Predicted}}\;$ is the mean of the predicted values, $\bar{\text{Observed}}\;$ is the mean of the observed values, S_Predicted_  is the standard deviation of the predicted values, S_Observed_ is the standard deviation of the observed values, and *m* is the number of independent variables.

In Table 3, we present the performances of EM and SOM ensembles by majority voting, CSPA, and HGPA. The results are provided for different numbers of clusters and their ensembles. From the results, it is found that, on average, SOM and EM ensembles by the use of the HGPA approach perform best, providing the highest rates of *R*^2^, PA, IA, MAE, and RMSE. The best accuracies are provided by ensemble size 3 (SOM2 × 4 + SOM3 × 3 + SOM3 × 4) for SOM and ensemble size 4 (*k* = 8, 10, 12, 13) for EM. In addition, majority voting has provided the lowest accuracy for EM and SOM ensembles in UPDRS prediction.

To evaluate the deployed methodology compared with previous methods in the literature, we performed several experiments on the PD dataset and presented the results in Table 4. The proposed method was compared with the SVR, ANFIS [87], MLR, HSLSSVR [88], neural network (NN), and DBN [89]. These perdition learning methods were compared with the HGPA + SOM + SVR ensemble and HGPA + EM + SVR ensemble as they provided better accuracy compared with other ensemble learning approaches. The results are provided for RMSE, MAE, and *R*^2^. The results reveal that ensemble learning methods, HGPA + SOM + SVR ensemble (Motor-UPDRS: MAE = 0.5540; RMSE = 0.4116; *R*^2^ = 0.9139; Motor-UPDRS: MAE = 0.5565; RMSE = 0.4179; *R*^2^ = 0.9058) and HGPA + SOM + SVR ensemble (Motor-UPDRS: MAE = 0.5594; RMSE = 0.4165; *R*^2^ = 0.9130; Motor-UPDRS: MAE = 0.5665; RMSE = 0.4186; *R*^2^ = 0.9018), can significantly impact the accuracy of both Total-UPDRS and Motor-UPDRS prediction. In addition, as shown in Table 4, it is found that clustering and dimensionality reduction techniques have significantly reduced the computation time of the proposed method for UPDRS prediction.

To assess the performance of the deployed method on the PD dataset with null values, we randomly considered 10% of patients' data as null values and predicted them with the SVD algorithm. The dense matrices are then used in EM and SOM for clustering and ensemble learning. We finally predict the UPDRS using the dataset with predicted values. The results are provided for HGPA + SOM + SVR ensemble and HGPA + EM + SVR ensemble in Figure 4. The results demonstrated that the SVD algorithm has been effective in null values prediction.

## 5. Discussion

Efficient detection of PD is crucial, as timely diagnosis and appropriate medication can delay the development of symptoms and difficulties resulting from this disorder [90]. Despite the significance of fast detection of PD, it is not an easy task because current detection measures are usually based on subjective indicators [91]. Besides, in the initial phases of PD, nonmotor signs, like depression, sleep disorder, and rapid eye movement, are more recognized than motor signs, which impacts the fast detection of the PD [92,93].

ML has been used for medical disease detection lately and particularly PD treatment [51]. This can be explained by the convenient performance and accurate results of ML techniques [94]. Classification of diseases is a significant type of predictive modeling. It is considered an important data mining approach because it clusters the population referring to a predetermined criterion. It is vital to compare the outcomes of various classification methods to decide which approach presents the best performance [95]. Hence, the main goal of this research is to assess several approaches that are utilized for PD prediction and classification. Even though ML methods have been assessed in several studies separately, the evaluation of these methods based on various datasets makes it complex to perform an accurate comparison among the deployed methodologies. Hence, it is vital to evaluate these methods in one comparative study based on a chosen dataset.

In this study, in the first step of data analysis, EM and SOM algorithms were implemented to produce various numbers of segments to have their ensembles for final clustering outcomes. Following that, the resulting clusters were used for ensemble learning UPDRS prediction by the SVR technique. Following that, the results are provided for different numbers of clusters and their ensembles. Referring to the outcomes, we can conclude that the performance of SOM and EM ensembles by the use of HGPA is the best among the deployed approaches based on *R*^2^, PA, IA, MAE, and RMSE measures. Besides, the evaluation of the proposed methodology in relation to previous methods in the literature was conducted based on various experiments on the PD dataset. The result of the deployed approach was compared with other approaches (SVR, ANFIS, MLR, HSLSSVR, and NN). Based on the findings, the HGPA + EM + SVR ensemble provided better accuracy compared with the other ensemble learning approaches.

## 6. Conclusion

Most of the presented methods for PD prediction depend strongly on human proficiency [96]. The benefits of deploying the ML in the medical sector are that they provide objective, context-independent, and data-driven analysis [97]. ML approaches have been utilized effectively in disease diagnosis and severity prediction [27,42,54,61,77–79,98–100]. Particularly, ML has also been utilized in analyzing the data collected from wearable IMU sensors for automated evaluation of motor disorders like PD [101–103]. Hence, the practical aim of this study entails providing supplementary, quick, and accurate methods that can aid experts in reaching more objective medical decisions considering the PD diagnosis. By deploying these methods in the appropriate systems, several gains can be acquired that entail reducing the expenses of manual diagnosis and minimizing diagnosis time.

Continuing this line of research and supporting previous literature, this study uses both unsupervised and supervised learning techniques to diagnose PD through UPDRS prediction. Besides, clustering, dimensionality reduction, and prediction learning techniques are used to create the PD diagnosis method. The basic aim of this paper is to conduct comparative research of the ML approaches for PD diagnosis. We concentrated on clustering and prediction learning methods to conduct the comparative study. Particularly, several clustering approaches for PD data segmentation and SVR ensembles to predict Motor-UPDRS and Total-UPDRS were used. The findings are then evaluated based on other prediction learning methods, MLR, neurofuzzy, and SVR techniques based on a real-world PD dataset. The finding of the study indicated the superiority of deploying EM with SVR ensembles in relation to decision trees, neurofuzzy and SVR combined with other clustering approaches in the prediction of Motor-UPDRS and Total-UPDRS.

Many previous works have been conducted focusing on patients' classifications, severity prediction, and remote monitoring. Still, there are future routes in each field to be investigated. Besides, several sensors such as magnetometer, accelerometer, and gyroscope have been utilized and assessed. Additionally, MRI, EEG signals, f-MRI, and DATSCAN images were utilized to present accurate predictions of the disease. Other research directions can be followed by utilizing other brain signal images such as ECG, EMG, and PCG. Other sensing modalities can be explored and combined to present a more accurate classification of the disease.

Even though ML methods in previous literature have presented high classification accuracy for PD detection, still, there are some obstacles related to feature extraction and selection which need to be addressed [104]. The utilization of several features can increase the computation time [105,106]. On the other hand, if fewer features were utilized, this will increase the complexity of extracting the features, which will accordingly impact the computation time. This paper has some shortcomings which should be considered in future research. The study is based on a real-world dataset to assess the proposed approaches, which has one limitation considering the number of features used in the prediction process. Other PD datasets with a larger number of features can be utilized in the evaluation of the deployed approaches. Large datasets can present more generalized outcomes. Emerging technologies can be used to collect data from patients using particular applications, as suggested by Bot et al. [107], in which the authors developed an application to collect the data from PD patients using their iPhones. This approach can ease the data collection from the public because of the availability of smartphones and help to present more generalizable outcomes. Furthermore, this study can be extended by incremental machine learning approaches to improve the computation time of previous PD diagnosis methods in processing large datasets [44,89].

## Figures and Tables

**Figure 1:** The proposed method for PD diagnosis.

**Figure 2:** SOM algorithm.

**Figure 3:** EM and SOM clusters.

**Figure 4:** Results of the method on predicted null values for UPDRS prediction.

**Algorithm 1:** Algorithm 1 PCA.

**Algorithm 2:** Algorithm 2 The procedure for missing value prediction by SVD.

**Table 1:** List of acronyms in this paper.

Acronyms	Description
AI	Artificial intelligence
ANFIS	Adaptive neurofuzzy inference system
ANN	Artificial neural network
CART	Tree classification and regression
CDSSs	Clinical decision support systems
CGP	Cartesian genetic programming
CSPA	Cluster-based similarity partitioning algorithm
CNN	Convolutional neural network
DBN	Deep belief network
DT	Decision tree
DSS	Decision support systems
DNN	Deep neural network
ebTL	Empirical Bayes transfer learning
ECG	Electrocardiogram
ELM	Extreme learning machines
EM	Expectation-maximization
EMG	Electromyogram
FDR	Fisher discriminant ratio
FNS	Fuzzy neural system
FOG	Freezing of gait
GA	Genetic algorithm
GRNN	Generalized regression neural networks
HGPA	Hypergraph partitioning algorithm
IMU	Inertial measurement unit
ISVR	Incremental support vector regression
K-NN	K-nearest neighbor
LR	Logistic regression
LSTM	Long short-term memory
LSVM	Lagrangian support vector machine
MAE	Mean absolute error
ML	Machine learning
MLP	Multilayer perceptron
MSA	Multiple system atrophy
MLP-LSVM	Multilayer perceptron-Lagrangian support vector machine
MLR	Multiple linear regression
NB	Naïve Bayes
NN	Neural network
NIPALS	Nonlinear iterative partial least squares
OPF	Optimum-path forest
PCA	Principal component analysis
PCG	Phonocardiogram
PD	Parkinson's disease
PSP	Progressive supranuclear palsy
RBM	Restricted Boltzmann machine
RF	Random forest
RBF	Radial basis functions
RNN	Recurrent neural network
RSSD	Sparse signal decomposition
RMSE	Root mean squared error
RBF	Radial basis functions
RNN	Recurrent neural network
RSSD	Sparse signal decomposition
RMSE	Root mean squared error
rTL	Regularized transfer learning
SOM	Self-organizing map
SVD	Singular value decomposition
SPECT	Single-photon emission computerized tomography
SVR	Support vector regression
SVM	Support vector machine
T-F	Time-frequency
UPDRS	Unified Parkinson's disease rating scale
WK	Wavelet kernel

**Table 2:** Previous literature on PD diagnosis.

Author(s)	Techniques																																					
	REG	SVM	FMCFW	CART	K-NN	NB	BT	RF	FNS	PCA	GSGP	GSGO	FDR	ANN	MLP	GRNN	EM	ANIFS	SVR	GA	WK	ELM	SOM	NIPALS	ISVR	MLP-LSVM	DNN	HMM	LASSO	CNN	rTL	ebTL	SVD	LSTM	RBM	LR	RNN	DBN
Nilashi et al. [46]																			√				√															√
Ghaderyan and Fathi [47]																																	√					
Paragliola and Coronato [48]																														√				√				
Balaji et al. [49]																																		√				
de Souza, et al. [50]																																			√			
Senturk [51]		√																																				
De Vos et al. [52]								√																												√		
Mohammed et al. [53]																														√								
Goyal et al. [54]																														√								
Xu and Pan [55]								√		√																												
Ribeiro et al. [56]																																					√	
Parziale et al. [57]																				√																		
Tsuda et al. [58]														√																								
Khoury et al. [59]		√		√	√	√		√																														
Çimen and Bolat [60]														√	√	√																						
Nilashi et al. [61]										√							√	√	√																			
Avci and Dogantekin [62]																				√	√	√																
Nilashi et al. [63]																							√	√	√													
Parisi et al. [64]																										√												
Prince and De Vos [65]	√							√																			√			√								
Zou and Huang [66]																													√		√	√						
Grover et al. [67]																											√											
Prashanth et al. [68]		√				√	√	√																														
Abiyev and Abizade [69]									√					√																								
Singh et al. [70]		√								√			√																									
Shetty and Rao [71]		√																																				
Ozkan [72]					√					√																												
Pahuja and Nagabhushan [73]		√			√									√																								
Rovini et al. [74]		√				√		√																														
Nilashi Ibrahim et al. [75]																		√															√					
Ashour et al. [76]		√												√																				√				

**Table 3:** SOM and EM ensembles by CSPA, HGPA, and majority voting for UPDRS prediction.

Ensemble size (SOM)	Ensemble technique	RMSE	MAE	IA	*P*A	**R**_**adjusted**_^2^
Motor-UPDRS						
2(SOM2 × 3 + SOM2 × 4)	CSPA	0.5980	0.4437	0.9208	0.9155	0.8999
	HGPA	0.5960	0.4416	0.9238	0.9200	0.9019
3(SOM2 × 4 + SOM3 × 3 + SOM3 × 4)	Majority voting	0.5720	0.4152	0.9306	0.9265	0.9078
	CSPA	0.5620	0.4150	0.9309	0.9266	0.9085
	HGPA	0.5540	0.4116	0.9335	0.9277	0.9139
4(SOM2 × 3 + SOM2 × 4 + SOM3 × 3 + SOM3 × 4)	CSPA	0.5772	0.4287	0.9283	0.9261	0.9067
	HGPA	0.5756	0.4286	0.9287	0.9263	0.9070
Total-UPDRS						
2(SOM2 × 3 + SOM2 × 4)	CSPA	0.6053	0.4463	0.9141	0.9101	0.8872
	HGPA	0.6016	0.4432	0.9166	0.9104	0.8928
3(SOM2 × 4 + SOM3 × 3 + SOM3 × 4)	Majority voting	0.5756	0.4269	0.9207	0.9173	0.9043
	CSPA	0.5700	0.4250	0.9230	0.9203	0.9043
	HGPA	0.5565	0.4179	0.9289	0.9240	0.9058
4(SOM2 × 3 + SOM2 × 4 + SOM3 × 3 + SOM3 × 4)	CSPA	0.5853	0.4395	0.9182	0.9138	0.8983
	HGPA	0.5799	0.4376	0.9193	0.9140	0.9026
Ensemble size (EM)	Ensemble technique	RMSE	MAE	IA	PA	**R**_**a** **d** **j** **u** **s** **t** **e** **d**_^2^

Motor-UPDRS						
2(*k* = 8,10)	CSPA	0.6122	0.4557	0.9103	0.9080	0.8904
	HGPA	0.5974	0.4521	0.9118	0.9092	0.8963
3(*k* = 8,10,12)	Majority voting	0.5897	0.4414	0.9149	0.9112	0.8998
	CSPA	0.5795	0.4397	0.9156	0.9117	0.9010
	HGPA	0.5789	0.4287	0.9173	0.9140	0.9028
4(*k* = 8,10,12,13)	CSPA	0.5623	0.4171	0.9257	0.9198	0.9049
	HGPA	0.5594	0.4165	0.9319	0.9254	0.9130

Total-UPDRS						
2(*k* = 8,10)	CSPA	0.6137	0.4574	0.9085	0.9049	0.8837
	HGPA	0.6086	0.4531	0.9092	0.9071	0.8848
3(*k* = 8,10,12)	Majority voting	0.5921	0.4480	0.9120	0.9081	0.8872
	CSPA	0.5912	0.4466	0.9135	0.9100	0.8904
	HGPA	0.5846	0.4398	0.9173	0.9101	0.8933
4(*k* = 8,10,12,13)	CSPA	0.5788	0.4370	0.9216	0.9180	0.8957
	HGPA	0.5665	0.4186	0.9281	0.9209	0.9018

**Table 4:** Methods' comparisons.

Method	Measure	MAE	RMSE	*R* ^2^	Computation time (ms)
NN	Motor-UPDRS	0.977	2.3836	0.7191	1072250
	Total-UPDRS	0.951	2.3135	0.7343	1043529
MLR	Motor-UPDRS	0.997	2.4142	0.6972	8953573
	Total-UPDRS	0.987	2.3911	0.7094	8845565
SVR	Motor-UPDRS	0.721	1.4942	0.8143	6743563
	Total-UPDRS	0.689	1.4526	0.8192	6633586
ANFIS	Motor-UPDRS	0.771	1.7047	0.7854	1534643
	Total-UPDRS	0.743	1.6062	0.7984	1525675
HSLSSVR	Motor-UPDRS	—	0.8158	—	—
	Total-UPDRS	—	0.8004	—	—
SOM + SVR	Motor-UPDRS	0.6340	0.5921	0.8518	538643
	Total-UPDRS	0.6421	0.6039	0.8421	535623
DBN	Motor-UPDRS	0.7645	1.6112	0.7914	974246
	Total-UPDRS	0.7321	1.5744	0.7996	964633
HGPA + SOM + SVR ensemble	Motor-UPDRS	0.5540	0.4116	0.9139	417435
	Total-UPDRS	0.5565	0.4179	0.9058	394352
HGPA + EM + SVR ensemble	Motor-UPDRS	0.5594	0.4165	0.9130	372223
	Total-UPDRS	0.5665	0.4186	0.9018	363422

## Data Availability

The data are freely available at https://archive.ics.uci.edu/ml/datasets.
